# Diagnosis of Retinal Diseases Based on Bayesian Optimization Deep Learning Network Using Optical Coherence Tomography Images

**DOI:** 10.1155/2022/8014979

**Published:** 2022-04-15

**Authors:** Malliga Subramanian, M. Sandeep Kumar, V. E. Sathishkumar, Jayagopal Prabhu, Alagar Karthick, S. Sankar Ganesh, Mahseena Akter Meem

**Affiliations:** ^1^Department of Computer Science Engineering, Kongu Engineering College, Perundurai, Erode 638060, Tamil Nadu, India; ^2^School of Information Technology and Engineering, Vellore Institute of Technology, Vellore 632014, Tamil Nadu, India; ^3^Department of Industrial Engineering, Hanyang University, Seoul, Republic of Korea; ^4^Renewable Energy Lab, Department of Electrical and Electronics Engineering, KPR Institute of Engineering and Technology, Coimbatore 641407, Tamil Nadu, India; ^5^Department of Artificial Intelligence and Data Science, KPR Institute of Engineering and Technology, Coimbatore 641407, Tamil Nadu, India; ^6^Department of Electrical and Electronic Engineering, Daffodil International University, Ashulia, Savar, Dhaka 1207, Bangladesh

## Abstract

Retinal abnormalities have emerged as a serious public health concern in recent years and can manifest gradually and without warning. These diseases can affect any part of the retina, causing vision impairment and indeed blindness in extreme cases. This necessitates the development of automated approaches to detect retinal diseases more precisely and, preferably, earlier. In this paper, we examine transfer learning of pretrained convolutional neural network (CNN) and then transfer it to detect retinal problems from Optical Coherence Tomography (OCT) images. In this study, pretrained CNN models, namely, VGG16, DenseNet201, InceptionV3, and Xception, are used to classify seven different retinal diseases from a dataset of images with and without retinal diseases. In addition, to choose optimum values for hyperparameters, Bayesian optimization is applied, and image augmentation is used to increase the generalization capabilities of the developed models. This research also provides a comparison of the proposed models as well as an analysis of them. The accuracy achieved using DenseNet201 on the Retinal OCT Image dataset is more than 99% and offers a good level of accuracy in classifying retinal diseases compared to other approaches, which only detect a small number of retinal diseases.

## 1. Introduction

Healthcare diagnosis is a primary focus area of deep learning research, with major industry players like GE Healthcare [1] investing heavily in it. Deep learning-based applications such as face recognition in phones, object recognition and detection, security systems, number plate detection, and a slew of other industrial applications have already gone commercial. These marketed applications are less vulnerable to errors and misclassifications than potential healthcare applications where mistakes might cost lives. As a result, accuracy in medical image analysis is critical in healthcare-based applications [2, 3], and focused research is required to make algorithms robust. In recent years, retinal diseases have become a severe public health concern. They develop slowly and without noticeable indications. Every year, millions of individuals throughout the world are diagnosed with retinal diseases, and these diseases express themselves in several ways. Retinal diseases may damage any area of the retina, causing vision impairments, and some can ultimately lead to blindness. Various retinal diseases include diabetic retinopathy (DR), macular pucker, glaucoma, macular hole (MH), age-related macular degeneration (AMD), drusen, central serous retinopathy (CSR), macular edema, vitreous traction, and optic nerve anomalies. These ailments lead to (i) loss of vision, (ii) floaters and cobwebs, (iii) flashing lights, (iv) objects seeming smaller or larger than they are, (v) decrease in peripheral vision or presence of shadows, and (vi) distortion of straight lines.

The term “prevention of retinal disease” refers to steps performed in advance to lessen the probability of vision loss, as well as the degree and effect of vision loss. In around 80% of instances, blindness and visual impairment may be prevented. A modest precautionary step can have a tremendous impact. Ophthalmologists often diagnose and treat retinal diseases. An ophthalmologist performs a full eye examination and searches for abnormalities everywhere in the eye. The Amsler Grid Test, OCT, Indocyanine Green Angiography, Ultrasound, Computed Tomography (CT), and Magnetic Resonance Imaging (MRI) are just a few of the procedures used to detect the location and severity of a disease. Among these, OCT is the most important screening tool for detecting rare retinal and optic nerve diseases, and three-dimensional retinal structural information is provided by OCT images using a light wave based approach [4]. Numerous researches have demonstrated that deep learning algorithms performed admirably when applied to medical image analysis for classification of skin diseases [5], cardiovascular diseases' risk prediction [6], lung cancer detection [7], and much more. These remarkable attempts encourage several studies to employ deep learning in diagnosing retinal diseases [8–11]. Since the introduction of deep learning techniques, OCT imaging has sparked a lot of interest in automated diagnosis for detecting a variety of retinal diseases [12]. But these studies were able to detect only a few types of retinal diseases such as Choroidal Neovascularization (CNV), Diabetic Macular Edema (DME), Drusen, DR, Glaucoma, AMD, CSR, MH [11, 13–20], and many more. Sample OCT images for a few retinal diseases and normal retina (without retinal disease) are presented in Figure 1.

Deep neural networks, notably the CNNs, are frequently employed in image classification tasks and have demonstrated substantial performance since 2012 [21–24]. CNN's study on medical image categorization has produced results that are comparable to those of human experts. CheXNet, for example, a 121-layer CNN that was trained on a dataset of over 100,000 frontal-view chest X-rays, outperformed the average performance of four radiologists. [25] provided a detailed overview of the uses of CNNs in medical image classification. Furthermore, previous attempts to classify and diagnose retinal diseases using OCT images have shown that standard deep architectures like VGGNet, DenseNet, and others may be ineffective because of their large parameter space. Transfer learning, on the other hand, might be a feasible strategy for dealing with enormous parameter spaces. Models can learn in one domain, where there is a lot of data, and then can transfer that knowledge to another domain, where there is not as much data. By leveraging previously trained models, we may train deep neural architectures that need a large number of learning parameters despite a low number of available images [26]. Deep learning models excel at learning from a large number of labeled cases [27], but they can only generalize to scenarios that were not seen during training. Overfitting and falling into a local optimum will occur when training samples are inadequate [28]. Furthermore, developing a deep learning model from scratch often needs a considerable amount of processing power and takes a long time. Transfer learning can help us in dealing with such scenarios. Another part of this research is that it applies Bayesian optimization to identify an ideal configuration for hyperparameters, as determining the best values for training CNN architectures is challenging. Hence, this work attempts to answer the following research questions:

  RQ1: will the presently available datasets be enough to detect a variety of frequently occurring retinal diseases?
  RQ2: how can pretrained CNN models be used to classify new datasets using transfer learning?
  RQ3: how can we customize the pretrained models? Does customization of such models significantly improve the quality of classification?
  RQ4: will the performance of the proposed models be improved by tuning hyperparameters appropriately?

The above research questions pave the way for classifying retinal diseases effectively. In this work, to address the above research questions, we developed a set of models using pretrained VGG16, DenseNet201, InceptionV3, and Xception architectures to automatically classify and detect retinal diseases from OCT images. To repurpose pretrained models, we use two strategies: freezing the convolution base (feature extractor) and training a few top convolution layers while freezing others (fine-tuner). Even though there have been more research attempts to identify retinal problems using CNN-based deep learning models, these studies have only tried to detect 3 to 5 types of commonly occurring retinal diseases from OCT images. In this work, we intend to build a few deep learning models that can detect seven different forms of retinal diseases, including AMD, CNV, DME, CSR, DR, Drusen, and MH. The developed models will categorize the OCT images as the normal or infected retina. We collected OCT images and divided them into eight categories to train and evaluate the models: seven for retinal diseases and one for normal. To the best of our knowledge, no work has addressed transfer learning with two fine-tuning processes combined with Bayesian Optimization for detecting a wide range of retinal diseases in the literature. The main contributions and novelty of this work can be summarized as follows:

- Providing an open-access dataset that contains OCT images (OCT Image Dataset) to help ophthalmologists in diagnosing diagnosis a wide range of retinal diseases by applying deep learning techniques
- Transfer learning is used in a novel way as a feature extractor and fine-tuner to build a few classifiers
- Tuning hyperparameters to find the optimal values using Bayesian Optimization (grid search, an exhaustive searching technique, has been used in the majority of the research studies to determine the ideal values)
- Exploring the transfer learning of pretrained CNNs with an optimum set of hyperparameters
- Analyzing the performance of the variants of pretrained CNNs through rigorous simulations
- A comparison of the performance of traditional and contemporary CNN architectures in terms of accuracy, precision, recall, and *F*1-score

We organize the rest of the article as follows: Section 2 discusses recent efforts relating to deep learning based retinal disease detection. In Section 3, we get into the intricacies of the dataset, deep neural network architectures, fine-tuning procedures, and Bayesian optimization. Experimental setup, adjusting the hyperparameters, and performance measures are discussed in Section 4. Following that, the experimental results and findings from the results are presented in Section 5. An in-depth analysis of error/misclassification of the images is also presented in Section 5. Finally, in Section 6, we summarize and conclude our study.

## 2. Literature Survey

The segmentation and thickness of retinal layers in OCT images are used to detect and diagnose retinal diseases. Changes in retinal layers owing to any disease are uncommon, and interpreting the data without a specialized benchmark technique is impossible. Standard image processing algorithms for detecting abnormalities in the retinal layer have certain drawbacks, such as being time-consuming and requiring sufficient subject knowledge. It is also challenging to generalize the procedure for automatic processing [29, 30]. With the evolution of technology and the introduction of Artificial Intelligence (AI), many researchers have begun to use deep learning based CNN to detect retinal diseases in OCT images. The application of CNN-based deep learning models is the topic of this review.

Obata [20] used deep learning and multivariate models to construct a model for predicting MH using preoperative OCT images and obtained precision of 46% and 40%, respectively. Hassan [18] used pretrained deep CNN to construct a system for reliable and automatic CSR detection from OCT images. For categorization, the authors used CNN models like AlexNet, ResNet-18, and GoogleNet. A statistical evaluation of parameters has been used to compare the performance of deep CNN, and AlexNet's classification accuracy from OCT Image Database was 99.64%. Subramaniam et al. [31] examined the most recent automated methods for detecting and classifying DR that used deep learning techniques. Binary classification, lesion-based classification, and vessel-based classification are some of the strategies used in this attempt. The publicly available fundus DR datasets have been provided, and deep-learning methodologies have been briefly explained. A work by [32] examined and analyzed the application of deep learning approaches at the various stages of DR detection using fundus images. This work included numerous parts of that pipeline, including widely used datasets, preprocessing approaches, and how they speed up and improve model performance, and the building of deep learning models for disease diagnosis and classification, as well as the localization of disease lesions.

The DeepDR system proposed by Dai [33] comprised three subnetworks: image quality evaluation, a subnetwork with lesion-awareness, and a grading subnetwork for DR. This system was trained on fundus images and used a multitask network with transfer learning. Venkatasen et al. [22] identified that, in a pooling layer, the positional relations have been suppressed in classical CNN. Since the positional information from images can be learned by a capsule network, the authors sought to apply OCT images on a capsule network to overcome this issue and found that a capsule network can be replaced by a capsule network and enhanced classification accuracy. This method attained a classification accuracy of 99.6%, which is comparable to other methods published for CNV, DME, Drusen, and normal images. In an attempt by [24], three types of retinal diseases, namely, CNV, DMD, and DME, have been classified. The hyperparameters, such as the number of epochs, size of each batch, and optimizer type, have been modified using random search optimization for better performance in classifying various retinal diseases. The accuracy of this method was 97.01%. In an attempt by [23], it diagnosed CSC using a deep learning model, which was able to use OCT images to discriminate chronic from acute CSC. The authors found that the performance was comparable to that of ophthalmologists and was better than VGG-16 and ResNet50. This model had a 93.8% accuracy rate for CSC diagnosis.

To classify retinal OCT images, Li et al. [34] developed a classification technique based on an ensemble of four classification model instances based on ResNet50. On the retinal OCT dataset, this study applied a 10-fold cross-validation procedure. The proposed technique was found to have a classification accuracy of 97.3%, which is comparable to ophthalmologists with substantial clinical experience. Huang et al. [35] developed a layer-guided CNN that can distinguish between a healthy retina and prevalent macular diseases including Drusen, CNV, etc. Specifically, retinal layer segmentation maps have been created using an effective segmentation network that can distinguish between retinal layers linked with relevant retinal lesions. LGCNN then combines the data from two lesion-related layers using two well-designed subnetworks. The precision was believed to be around 88%. [13] suggested a deep learning based classifier for computer-assisted categorization of DME, Drusen, and CNV. This study used a six-layer deep CNN to perform the classification of the OCT images into four types, achieving an accuracy of 99.69%. [16] showed that utilizing a Generative Adversarial Network (GAN) to perform few-shot learning can increase the applicability of deep learning in OCT diagnosis of uncommon diseases. Four major classes with a large number of datasets and five classes of rare retinal diseases with a few-shot dataset have been considered for this study. The accuracy of this approach was 93.9%. [36] described a deep CNN architecture for effectively identifying and classifying patients into normal, DMD, and DME categories. The Kuan filter is used to remove speckles from raw OCT images to reduce intrinsic speckle noise. The classification accuracy of this work has been 95.7%. [11] used DenseNet-100 as a feature extractor, with CenterNet as a one-stage detector for localizing and classifying disease lesions. The authors tested the technique on two datasets, APTOS-2019 and IDRiD, and found that it had an average accuracy of more than 97%. While reviewing the present works, we find a work by Kaliappan et al. [19] that presented OCT images collected from the King Abdullah University Hospital in Irbid, Jordan. CNV, MH, CSR, Geographic atrophy, Macular Retinal Oedema, and Vitreomacular Traction are among the eye diseases by this collection, which includes 21,991 OCT images. A model based on the U-Net has been built to categorize where the images are of real Jordanian patients, and the annotation was done by ophthalmologists. This dataset was subjected to two classification tasks: a binary classifier that distinguishes between images from healthy eyes and diseased eyes (abnormal). The binary categorization was 84.9% accurate. Multiclass classification is the second classification challenge, in which the model is trained to discriminate between several diseases in addition to the normal condition, with 63.68% accuracy. In addition, a summary of existing deep learning models in glaucoma assessment utilizing OCT images has been provided by [14]. Apart from using deep learning models, image segmentation techniques and algorithms based on machine learning have also been proposed for image analysis [37–41].

As seen from the research attempts described above, deep learning architectures are increasingly being used in the diagnosis of retinal diseases from OCT images. However, various gaps in the usage of deep learning architectures that must be addressed include faster training times and fewer parameters. We employ transfer learning to reduce training time, and the optimal values for hyperparameters are chosen using Bayesian Optimization. Furthermore, we found that the current research works sought to detect 3 to 5 retinal diseases. We collected OCT images with AMD, CNV, DME, CSR, DR, Drusen, and MH diseases and made them publicly available to find a wide variety of retinal abnormalities.

## 3. Materials and Methods

The purpose of this study is to develop and compare a few models for diagnosing retinal diseases using OCT images using various CNN architectures. This section discusses all of the materials as well as the procedures used.

### 3.1. Datasets

The OCT images for retinal diseases acquired from Kaggle fall into the following categories: AMD, CNV, DME, DRUSEN, and NORMAL. We have also used images from OPEN-ICPSR, a no-cost, self-publishing resource for social, behavioral, and health sciences research data, to add a few more retinal diseases like CSR, DR, and MH. The OCT images collected from various sources such as Kaggle and Open-ICPSR are then augmented. Both datasets contain different classes and different numbers of images. To use this as input to a neural network model, the datasets have to be equalized. The greater the amount of data available to the network, the more features it will be able to learn. Image augmentation is a technique for artificially producing new training images. Rotation, flipping, cropping, and translation are examples of image augmentation techniques that have been used to assist lessen a model's overfitting. The dataset comprises around 24,000 images after augmentation, approximately 3000 images in each category. After equalizing the data from both datasets, a new dataset called “Retinal OCT–C8” is developed and hosted as a public dataset on Kaggle. We have also used on-the-fly data augmentation to deliver real-time augmentation. That is, while a model is still being trained, it generates augmented images on the fly and ensures that each epoch of the model receives new variants of the images. The images that have been altered are not included in the original image corpus. If this was the case, the model would be continually exposed to the original images, leading to overfitting. Normalization of the image's size and format is a critical operation. All images have been resized to 224 *∗* 224 (for VGG16 and DenseNet201) and 299 *∗* 299 (for InceptionV3 and Xception) pixels at a resolution of 96 *∗* 96 dots per inch.

### 3.2. CNN

CNN architecture is a popular deep learning method for image classification and a key technique for modeling complex processing in applications with a lot of data. It is cutting-edge in image classification tasks and is programmed to extract visual patterns from input images directly. CNN is based on the work of Kunihiko Fukushima, a Japanese scientist who invented the Neocognitron, a very primitive image recognition neural network. The challenge of handwritten digit categorization has been effectively implemented by CNN with a gradient-based algorithm. It then became the state-of-the-art in a variety of object recognition tasks, and it is currently utilized in a variety of other fields, including object tracking and identification and text and action recognition. A significant property of CNN is its capacity to automatically learn hierarchical feature representations. Edge-based features are often detected by the first few layers of CNN. The early layers' output is sent into intermediate layers, which extract more complicated features like corners and edges. The layers recognize higher-level features like objects, faces, and so on as we progress deeper into the network. This means that the earliest layers' features are generic and can be used to solve a range of issues, but the latter layers' characteristics are particular to the dataset and task at hand. When compared to traditional feed-forward neural networks, CNN has the advantage of requiring fewer neurons and hyperparameters. For image recognition applications, several baseline CNN architectures have been created and effectively utilized to complex visual imagery problems. To develop the proposed models in this work, we used pretrained models including VGG16, DenseNet201, InceptionV3, and Xception. In the next section, we will go over these ground-breaking CNN designs.

### 3.3. VGG16

VGG16 is a 16-layer network presented in 2014 by Simonyan and Ziserman of Oxford University's Visual Geometry Group Lab [28], It is much deeper than AlexNet but has a simpler network, because huge kernel-size filters are replaced with multiple 3 *∗* 3 kernel-size filters. VGG16 is made up of thirteen convolutional layers and three fully connected layers.  Figure 2 depicts the architecture of VGG16. VGG19, an improved version of VGG16, has sixteen convolutional layers and three fully connected layers.

### 3.4. DenseNet201

DenseNet201 [42] is a CNN that employs dense blocks to establish dense connections between layers, with all levels being linked directly. Each layer in a feed-forward technique is linked to every other layer. When a layer is generated, the feature maps of all previous layers are regarded as independent inputs for each layer, whereas the feature maps of the current layer are passed on as inputs to all subsequent layers. The elimination of the vanishing-gradient problem, improved feature propagation, feature reuse, and a large reduction in the number of parameters are all advantages of DenseNets. For these reasons, we chose to create a model using this CNN variation.  Figure 3 depicts a dense 5-layer block.

### 3.5. Inception

InceptionV1 is a deep convolutional architecture that was launched as GoogLeNet by [43]. The Inception design was later modified in several ways, the first of which was the addition of batch normalization [44]. This is named InceptionV2. InceptionV3 [45] includes label smoothing, factorized 7 × 7 convolutions, and a classifier for transferring label information deeper down the network. The model's symmetrical and asymmetrical building components include convolutions, max pooling, concerts, dropouts, and fully connected layers. The softmax function is part of the InceptionV3 architecture's last layer, which includes 48 layers in total and an input layer that accepts images with a resolution of 299 × 299 pixels. While preserving speed and accuracy, InceptionV3 considerably cuts processing expenses.

### 3.6. Xception

Xception is a variation of the Inception architecture that uses depth-wise separable convolutions instead of the standard Inception modules. The Xception architecture [46] has 36 convolutional layers as its feature extraction base and except for the first and last layers, the convolution layers are divided into 14 modules, each of which is surrounded by linear residual connections. In a nutshell, the Xception architecture is a residually connected depth-wise separable convolution layer stack. This model substituted depth-wise separable convolutions for standard inception modules, which were preceded by a point-wise convolution (1 *∗* 1). In most traditional classification problems, the Xception architecture outperformed VGGNet, ResNet, and InceptionV3.

### 3.7. Transfer Learning

Transfer learning has recently piqued the interest of researchers. It is an approach for fine-tuning previously trained neural networks to create new AI models [47]. In other words, it uses established knowledge to address distinct but similar domain issues. Its goal is to complete information transmission between related areas, and it has become extremely popular because it cuts training time and utilizes far fewer data to increase performance. Transfer learning is typically portrayed in computer vision through the use of pretrained models. A pretrained model has been trained on a large benchmark dataset to handle a problem similar to the one at hand. Importing and using models that have previously been tested and published is one technique to reduce the computational expense of training new models (e.g., VGGNet, Inception, and Exception). Canziani et al. [48] used the ImageNet dataset to investigate the performance of pretrained models on computer vision challenges. Using transfer learning, large CNNs are used to train several pretrained models. We repurpose the pretrained CNN versions VGG16, DenseNet201, InceptionV3, and Xception for our dataset by removing the classifier and adding a few classification layers, as well as retraining the top layers of convolution base. Here is what they are:

  Training the classifier (feature extractor) by freezing the convolutional base: we can preserve the convolution base in its original form while using ImageNet weights. The classifier produces 1000 different output labels in pretrained models; however, the number of neurons in the output layer can be determined by the number of classes in our dataset. As a result, we may import the convolutional base and add our classifier to it. The classifier receives the output from the convolutional base. The pretrained model can be used as a feature extractor in this approach.
  Fine-tuning a few top layers: we maintain the weights of the initial layers frozen and retrain the higher layers to learn the dataset-specific features since the lower layers correspond to general features (dataset independent features) and the higher layers refer to unique features (dataset dependent features). Pretrained models are used as a fine-tuner in this case.

Since the pretrained models trained on ImageNet have been used to identify retinal syndromes in many of the attempts described in Section 2, we also employ transfer learning to fine-tune our models using the above two ways. Even though we have roughly 24000 OCT images for training and testing the models, this may not be enough for deep neural networks, resulting in overfitting. When the target data set is tiny, the main benefit of transfer learning becomes apparent. The model may be prone to overfitting in many circumstances, and augmentation may not necessarily solve the overfitting problem. As a result, transfer learning has been deployed. We can also save a substantial amount of training time by relying on existing knowledge because the weights learned from ImageNet datasets have been used. Retraining a model from scratch demands the random selection of all weights, which takes huge computational power and time. Hence, training the classifier and the convolution base's top layers should be sufficient. Here is a rundown of the transfer learning techniques employed in this study:

- Pick one model at a time from the list of pretrained models
- Add classification layers according to the dataset and pretrained models
- Train the model using strategies 1 and 2 in turn
- Out of all the pretrained models, find the strategy with the highest accuracy

The details and results of implementing these strategies are discussed in Sections 4 and 5.

### 3.8. Hyperparameters Optimization

Hyperparameters are network parameters that define the structure of the network, such as the hidden units' size, dropout, activation function, and weight initialization, as well as how the network parameters such as learning rate, momentum, batch size, and epochs are trained. The process of identifying the best settings for hyperparameters in a learning algorithm is known as hyperparameter tuning. Hyperparameter tuning is to identify optimal values for hyperparameters to reduce the loss function and improve results. The various optimization techniques include manual search, grid search, random search, and Bayesian Optimization. A random search produces hyperparameter combinations at random, tries to fit the dataset, and assesses its accuracy. It is possible that certain configurations that would have been ideal were overlooked. While random search is quicker, it may not always produce the best results. In manual search, using previous experience, we select hyperparameters for a model. The model is then trained and evaluated using these parameters. This approach is repeated with a different set of values for the same hyperparameters until maximum accuracy is acquired or the model has attained the optimal error. Because manual search is biased and comprehensive, it may not be the best option. In grid search, the same procedure as random search is used for tuning the hyperparameters, but with one exception. Each hyperparameter combination is tried. This adds time to the process and makes it inefficient. However, it is the most successful since the best option is less likely to be overlooked.

Unlike grid and random searches, Bayesian optimization takes advantage of previous iterations of the algorithm. Each hyperparameter guess is independent in the grid and random searches. With Bayesian techniques, on the other hand, we move closer to the perfect solution with each selection and testing of alternative hyperparameters [49, 50]. When it comes to identifying the optimum potential hyperparameter settings, Bayesian optimization algorithms surpass grid and random searches. Because of the amount of data and computing density, more time is needed to train deep learning models. Bayesian optimization can be quite useful in these situations. In this work, we employ Bayesian optimization to optimize the hyperparameters of the classifier layers in conjunction with pretrained models. To summarize, we suggest using CNNs powered by transfer learning and Bayesian optimization to create a few models to classify OCT images. The workflow of the proposed models is depicted in Figure 4. A few classifiers have been developed using the pretrained models and retrained using transfer learning for feature extraction. While fine-tuning, optimum number of convolution base layers to be retrained has been found. The ideal values for hyperparameters have been determined via Bayesian optimization. For the set of values of hyperparameters, the pretrained models have been trained using the training dataset and stored as checkpoints. The models with the ideal hyperparameter values that provided the highest accuracy have been evaluated using the validation dataset. Finally, using the testing dataset, the performance of classifiers is assessed.

## 4. Details of Experiments

We conducted two sets of experiments, namely, Feature Extractor and Fine-tuner, to examine the performance of the models developed, and the details of experiments are given below.

### 4.1. Experimental Platform

We imported the necessary Keras model architectures and instantiated them with ImageNet weights. Since the developed models consume a lot of power and require high-performance hardware to function properly, we ran the proposed models on Graphical Processing Units (GPUs). The hardware and software configurations utilized are listed in Table 1.

### 4.2. Tuning of Hyperparameters

In deep learning algorithms, hyperparameters are significant because they specify training details and have a direct impact on model output [51]. Choosing the appropriate hyperparameter settings is critical. We have used Bayesian Optimization to obtain the best values for hyperparameters while maintaining excellent accuracy in this study. It is a method for determining the lowest or maximum of an objective function. In this study, we wish to maximize the accuracy and use the Gaussian Process (GP) as the probabilistic model [50]. GP generates a hypothesis for unknown parameters based on previously known parameters. Although the Bayesian approach takes longer to select hyperparameters, it takes less time to assess the objective function, resulting in low computational costs.  Table 2 summarizes the hyperparameters tuned in our work, as well as their search space.

### 4.3. Experimental Setup

After the dataset has been randomized, the training and testing datasets have been split, with 70% of the dataset being used to train the classifier, 15% being used for validation, and 15% being used for testing. This is done to guarantee that as much data as possible is available for training, resulting in a more accurate model. The training and validation datasets have been used to train and fit the model, while the test set has been used to evaluate the model's prediction performance on samples it had never seen before. For both sets of experiments, we downsized all images to 224 *∗* 224 *∗* 1 and 299 *∗* 299 *∗* 1 and used in-place image augmentation to accommodate the input of the developed models. In all of the models, the categorical cross-entropy is employed as the loss function. We ran the models for 75 epochs but stopped them early. Early stopping is a technique, in which the model is trained for an arbitrary number of epochs and then stopped when the validation accuracy or validation loss does not improve. To monitor the validation accuracy, we employed early stopping and set patience to 5, which helps quit the training if the validation accuracy does not improve. Another reason for early stopping is that it allows us to terminate the training process when the model becomes overfit. To conduct the proposed tests, we removed the classifier layer from these models and replaced it with our own. For each of the pretrained models, Table 3 shows the number of fully connected layers added to the classification block.

The actual output layer in all of the pretrained models is a 1000-class softmax activation. This layer is replaced with an eight-category softmax layer. The number of neurons in each fully connected layer is a configurable hyperparameter. Pretrained models such as VGGNet, DenseNet201, InceptionV3, and Xception have been utilized as feature extractors in the first set of tests, and the retrieved features have been then used to train the newly added classifier. The weights learned from the ImageNet dataset have been used in the convolution base. In the second set of tests, we retrained a few top layers of the convolution base. Bayesian optimization has been used to find the best values for the hyperparameters. A total of 20 iterations of Bayesian optimization have been performed. We set the number of epochs to 75 for each iteration of Bayesian optimization. Each iteration's accuracy and loss have been recorded.  Table 4 shows the hyperparameter settings that resulted in the highest accuracy for all models. The hyperparameters found within 20 iterations were deemed best in our study because more iterations did not result in substantial changes. If we employ a vast search space, we can get a better set of values for hyperparameters, but at the expense of a huge computation time.

### 4.4. Performance Metrics

Following the development of the models, the next step is to evaluate their effectiveness using metrics against the test datasets. The developed CNN models have been evaluated using a variety of performance measures, including accuracy, precision, recall, *F*1-Score, macro, and weighted average. True Positive (TP), True Negative (TN), False Positive (FP), and False Negative (FN) indices have been used to calculate the values for the performance metrics. TP stands for the total number of correctly classified images in each class. FP stands for the number of images misclassified in all other classes except the correct one. FN stands for the number of images misclassified in the relevant class. The number of images correctly identified in all other classes except the correct one is referred to as TN. Equations (1) to (4) are used to determine TP, FP, TP, and TN, with *i* = 1,2,3, and 4 signifying the four classes.

(1) $$\begin{array}{c} tp_{i}=\;c_{ii}, \end{array}$$

(2) $$\begin{array}{c} fp_{i}=\;\overset{n}{\underset{l=1}{\sum }}\left(c_{li}\right)-tp_{i}, \end{array}$$

(3) $$\begin{array}{c} \;fn_{i}=\;\overset{n}{\underset{l=1}{\sum }}\left(c_{il}\right)-tp_{i}, \end{array}$$

(4) $$\begin{array}{c} tn_{i}=\;\sum_{l=1}^{n}\sum_{k=1}^{n}\left(c_{lk}\right)-tp_{i}-fp_{i}-fn_{i}. \end{array}$$

Accuracy is defined as the number of samples properly identified as belonging to a specific class divided by the total number of samples in that class and is calculated by

(5) $$\begin{array}{c} \text{accuracy}=\frac{\left(\text{TP}+\text{TN}\right)}{\left(\text{TP}+\text{TN}+\text{FP}+\text{FN}\right)}. \end{array}$$

The number of samples correctly categorized as a certain class out of the total number of actual samples in that class is defined as recall and is computed using

(6) $$\begin{array}{c} \text{recall}=\frac{\left(\text{TP}\right)}{\left(\text{TP}+\text{FN}\right)}. \end{array}$$

Precision is defined as the number of samples accurately categorized as a specific class out of the total number of samples categorized as that class and is given by

(7) $$\begin{array}{c} \text{precision}=\frac{\text{TP}}{\left(\text{TP}+\text{FP}\right)}. \end{array}$$

*F*1-Score is defined as the harmonic average of the precision, and recall, that is, the weighted average of Precision and Recall. It is calculated as in

(8) $$\begin{array}{c} \text{F}1-\text{score}=\frac{\left(2*\text{precision}*\text{recall}\right)}{\left(\text{precision}+\text{recall}\right)}. \end{array}$$

The unweighted average of the class-wise scores is used to determine the macro average. To get the final averaged metric, macro-average gives equal weight to each of the eight classes in the dataset. The weighted average is computed by taking the weighted average of class-wise scores, with the weights proportional to the number of instances of each class; that is, the contribution of each class to the average is weighted by its size.

## 5. Experimental Results and Findings

We examined the performance of the pretrained CNN models used in this study, including VGG16, DenseNet201, InceptionV3, and Xception, as feature extractors and fine-tuners. The experiments have been conducted with the tuned hyperparameters listed in Table 4, which generated the good results during training. The classification report for the proposed models is presented in Tables 5–8. Due to the uncertain nature of images, the models may result in better accuracy but fail to realize the images properly and hence may perform poorly when the images are varied. This indicates that the models are not robust enough and hence limit their usage. So, accuracy is not enough alone for classification task. We need to look at some other metrics to make sure our models are reliable. Because the number of images in each class in the test data set is roughly similar, the weighted and macro averages for each model are nearly identical.

Table 9 provides a comparison of the performance of the models developed in this work.

Since we need to classify retinal diseases into one of eight categories, we assess the performance of all the models in the dataset against each of the eight classes. For this, we utilized equations (1) to (4) to calculate the indices TP, FP, TN, and FN. We use the confusion matrix obtained during testing to calculate the values of these indices. As we all know, the confusion matrix is a visualization tool to know how well-predicted classes match the actual classes. The confusion matrix acquired when testing VGG16 is shown in Figure 5. The diagonal elements represent correct classifications. On the other hand, the rest are misclassifications. The *X*-axis depicts predicted classes, whereas the *Y*-axis depicts actual classes. For example, VGG16 predicted 20 images with DME disease as CNV, 1 DME image as AMD, and so on, as shown in Figure 5(a).

### 5.1. Performance Comparison with Other Models

The performance of the models developed in this work is further evaluated by comparing them to other similar models that categorize retinal diseases. The comparison results are summarized in Table 10.

From Table 10, we can see that the test accuracy of the proposed models is relatively good compared with the accuracy of other recent deep learning methods. One good thing about the proposed models is that they all attempt to identify more retinal diseases from OCT images than with other approaches.

## 6. Results and Discussion

Table 9 presents the overall validation and testing accuracy for each of the models across all eight classes. As shown in Table 9, when employing the pretrained models as feature extractors and training the classifier using the extracted features, the validation and testing accuracy is lower than that when retraining a few top layers. The fine-tuning technique keeps the pretrained models' weights on earlier levels and retrains them on the top layers. But, in strategy 1, the pretrained models have been just employed as feature extractors, with no fine-tuning, and the top layers are not retrained exclusively for our dataset. As a result, the features learned are unique to ImageNet, and so the accuracy is lower than strategy 2. But, interestingly, the three models DenseNet201, InceptionV3, and Xception achieved high accuracy for strategies 1 and 2, showing that optimization allowed for improved generalization in these models. VGG16, on the other hand, comparatively has low accuracy. We may be able to improve accuracy by retraining this model for more epochs. We stopped training the models since we employed early stopping, and there was no change in validation accuracy after 5 iterations. We experimented by removing early stopping and found that there is an increase in accuracy in VGG16 as well. While analyzing the reason for the high accuracy of DenseNet201, we found that better feature reusing capability leads to high accuracy. In addition, DenseNet201 alleviates the vanishing-gradient problem, supports feature propagation, and substantially reduces the number of parameters. Nevertheless, this model requires a large amount of GPU memory for convolution operation. Based on our review of the literature, we found that a few attempts used GPUs to train the models. But we are unable to compare the performance of the proposed models with these models in terms of training time due to the differences in GPU configuration and disparity in the datasets. Because we retrain a few top layers of the models in addition to the classifier component, training as feature extractors takes less time than training as a fine-tuner. This clearly indicates that retraining the entire model would take much more time. Hence, it is evident that transfer learning reduces the training time. Among the developed models, even though DenseNet201 gives the highest accuracy, it takes huge time to train the models, as it has a huge number of layers. We further calculated the number of parameters retrained in each of the developed models, and the results are presented in Table 11.

Among all the models, DenseNet201 retrained a smaller number of parameters. Nevertheless, the time taken by this model for training is large as it has a huge number of layers. We enumerated a set of research issues to be addressed by the proposed effort in Section 1. Now, we will take a look at how the proposed models have addressed these issues. In this attempt, four pretrained models trained on the ImageNet dataset have been used to develop models for detecting retinal diseases from OCT images. These pretrained models are simple to use and produce better results with less training effort because they provide the architecture for free. During transfer learning in the proposed study, the pretrained models have been deployed with a few alterations on a new classification task. This resulted in higher accuracy than constructing models from the ground up. Table 10 shows how this works. Using fine-tuning, we can use pretrained networks to recognize classes in new datasets that they were not trained on before. Fine-tuning was more accurate than transfer learning via feature extraction because the weights of the later layers were retrained on the dataset used in the study. Bayesian optimization was then used to find the ideal values for the hyperparameters, which resulted in a considerable improvement in performance overutilizing the default values for the hyperparameters. To summarize, we believe that the following factors, when compared to other models, contribute to improved accuracy.

- Finding optimal values for the hyperparameters via Bayesian optimization
- Using transfer learning to fine-tune the top layers of the convolutional base

### 6.1. Error Analysis

To understand the challenges of this task, we carried out further analysis of the errors made by our models. Error Analysis refers to the process of examining test set images that the models misclassified so that we can understand the underlying causes of the errors. A classification model's results on new images can be categorized into one of four categories, namely, true positives, false positives, true negatives, and false negatives. True or false refers to whether the predicted class matches the actual class in all four cases, and positive or negative refers to the classification the model has assigned to observation. For instance, in the confusion matrix for the VGG16 model, we can find that the true positive for the AMD class is 336. This indicates that out of 350 AMD samples, 336 samples have been classified as AMD, and 14 instances have been misclassified not AMD. Similarly, for CNV, only 244 instances have been classified correctly as CNV, and 106 instances have been misclassified as not CNV. Below we discuss a few cases.  Figure 6 shows an OCT image of CNV retinal disease and a normal image.

The actual class for the image in Figure 6(a) is CNV. But the VGG16 model has predicted this image as normal, that is, without any retinal disease. Although the feature map strongly highlights the presence of symptoms for retinal disease, we cannot immediately be sure that this is the reason for misclassification. But the image is correctly classified by other models. Similarly, an OCT normal image has been predicted by VGG16 as having CNV disease. One reason may be that the VGG16 model has not fetched the features from the images properly. So, the details that led to the misclassification must be found. As a result, we believe that the misclassification data can be used to increase classification accuracy. Assume that images are frequently misclassified with many classes for one single class. Instead of considering all image classes, we should focus on specific misclassified classes to mine important information.

## 7. Conclusion and Future Work

Retinal diseases have become a major public health concern in recent years and accurate detection is a challenge. Manual localization of retinal disease requires the use of trained human experts to detect finer points of interest in OCT images and classify them into the relevant disease using a grading system. Automated retinal disease detection models are necessary to overcome the obstacles of manual detection, and this work investigated the application of deep learning models to diagnose retinal diseases using OCT images. Transfer learning has been chosen for this research because it has the following advantages: (i) no need for excessively large training datasets; and (ii) only the weights of a few top layers need to be retrained, requiring little processing effort. Since developing a model from scratch requires a lot of computational power, we used pretrained models, such as VGG16, DenseNet201, InceptionV3, and Xception as feature extractors and fine-tuners.

With exception of VGG16, all other models showed comparable accuracy to other deep learning models, when using them as classifiers. When fine-tuned, however, they achieved an accuracy of over 95%. Because DenseNet201 is the deepest of all the pretrained models used in this study, it takes longer training epochs to achieve high accuracy. Additionally, Bayesian optimization was used to select the best values for hyperparameters used during training. The findings of this study led us to believe that using pretrained models based on Bayesian Hyperparameter optimization and transfer learning for the classification of retinal diseases from OCT images is a promising alternative. As a result, this research can be extended to detect a variety of additional retinal diseases and construct a few more deep learning models with fewer parameters and less training time. There is a trade-off between the selection of hyperparameters and the training time. Hence, we plan to further explore hyperparameters used in the optimization process. In the meantime, the trained model could be used with mobile devices to assist health practitioners to make fast and precise decisions about retinal diseases.

## Figures and Tables

**Figure 1:** Sample OCT images. (a) AMD. (b) CNV. (c) CSR. (d) DME. (e) DR. (f) Drusen. (g) MH. (h) Normal.

**Figure 2:** VGG16 architecture.

**Figure 3:** A 5-layer dense block [43].

**Figure 4:** Workflow for the proposed classifiers.

**Figure 5:** Confusion matrix. (a) VGG16 (feature extractor). (b) VGG16 (fine tuner).

**Figure 6:** Error analysis. (a) An OCT image with CNV disease. (b) An OCT normal image.

**Table 1:** Experimental platform.

Item name	Specifications
GPU	GPU DELL EMC 740
RAM	128 GB
GPU RAM	32 GB
DISK	4 TB
OS	Ubuntu
Language	Python
IDE	Jupyter notebook environment

**Table 2:** Hyperparameters and their search space.

Parameter	Search space	Description
Optimizer	Adam, RMSProp, SGD, AdaDelta	To optimize the input weights by comparing the prediction and the loss function
Learning rate	1*e* − 3, 1*e* − 4, 1*e* − 5, 1*e* − 6	To determine the step size at each iteration while minimizing the loss function
Activation function	ReLu, Elu and Tanh, Leaky ReLu	To introduce nonlinearity into the output of neurons
Number of neurons in customized layers	64,128, 56, 512,1024	To compute the weighted average of the input
Batch size	32,64,128	Number of training examples utilized in one iteration

**Table 3:** Modification of the classification block.

Pretrained models	Number of layers added
VGG16	2 fully connected + 1 softmax
DenseNet201	2 fully connected + 1 softmax
InceptionV3	1 fully connected + 1 softmax
Xception	1 softmax

**Table 4:** Hyperparameters with tuned values.

Hyperparameters	VGG16		DenseNet201		InceptionV3		Xception	
	Feature extractor	Fine-tuner	Feature extractor	Fine-tuner	Feature extractor	Fine-tuner	Feature extractor	Fine-tuner
Optimizer	Adam	Adam	Adam	Adam	RMSProp	RMSProp	Adam	Adam
Learning rate	0.0001	0.0001	0.00001	0.00001	0.00001	0.0001	0.001	0.0001
Activation	tanh	tanh	elu	relu	tanh	relu	elu	relu
No. of neurons	256	512	128	128	64	512	128	256
Batch size	32	32	32	32	32	32	32	32

**Table 5:** Performance of VGG16.

Class labels	Precision (%)		Recall (%)		F1-score (%)	
	Feature extractor	Fine tuner	Feature extractor	Fine tuner	Feature extractor	Fine tuner
AMD	99.41	100	96	99.71	97.67	99.86
CNV	79.74	87.24	69.71	95.71	74.39	91.28
CSR	83.05	97.77	96.57	100	89.3	98.87
DME	73.83	93.49	62.86	90.29	67.90	91.86
DR	81.44	99.14	84	99.14	82.7	99.14
Drusen	67.19	95.72	60.86	83.14	63.89	88.99
MH	95.41	100	77.14	98.29	85.31	99.14
Normal	62.65	89.81	87.71	95.71	73.1	96.67
Macro average	80.34	95.4	79.36	95.25	79.28	95.23
Weighted average						

**Table 6:** Performance of DenseNet201.

Class labels	Precision (%)		Recall (%)		*F*1-score (%)	
	Feature extractor	Fine tuner	Feature extractor	Fine tuner	Feature extractor	Fine tuner
AMD	97.34	100.00	94.82	100.00	95.12	99.12
CNV	91.08	99.82	92.45	98.12	92.91	89.66
DME	94.26	99.55	89.12	99.34	90.72	99.61
CSR	97.18	99.11	93.29	97.56	94.61	98.55
DR	89.99	99.79	96.51	98.69	94.95	97.99
Drusen	91.73	99.51	93.21	98.88	92.91	97.99
MH	91.00	100.00	96.57	99.11	93.98	98.44
Normal	92.09	99.91	94.12	98.99	94.01	98.03
Macro average	93.08	99.71	93.76	98.84	93.65	97.42
Weighted average	93.08	99.71	93.76	98.84	93.65	97.42

**Table 7:** Performance of InceptionV3.

Class labels	Precision (%)		Recall (%)		*F*1-score (%)	
	Feature extractor	Fine tuner	Feature extractor	Fine tuner	Feature extractor	Fine tuner
AMD	90.12	95.62	91.81	92.31	90.60	93.27
CNV	88.15	96.71	90.81	95.91	87.96	90.06
DME	90.31	93.98	87.48	93.27	87.72	91.72
CSR	88.18	95.91	91.02	91.78	90.34	89.45
DR	87.99	93.11	90.18	93.91	90.06	91.62
Drusen	89.41	96.81	89.38	89.95	89.43	93.02
MH	90.01	96.21	91.64	96.81	89.23	91.62
Normal	88.62	95.47	89.74	95.99	90.82	93.49
Macro average	89.10	95.48	90.26	93.74	89.52	91.78
Weighted average						

**Table 8:** Performance of Xception.

Class labels	Precision (%)		Recall (%)		*F*1-score (%)	
	Feature extractor	Fine tuner	Feature extractor	Fine tuner	Feature extractor	Fine tuner
AMD	92.17	98.23	89.23	98.56	90.12	96.99
CNV	90.56	98.18	91.10	97.34	90.06	95.61
DME	89.91	96.99	88.97	98.13	89.97	97.03
CSR	88.65	97.26	90.45	96.99	91.22	98.41
DR	92.11	98.61	89.34	95.09	90.23	96.21
Drusen	91.99	97.49	92.31	95.01	91.24	95.24
MH	92.05	98.12	91.81	96.38	90.03	95.02
Normal	90.51	94.78	89.45	95.73	91.45	96.12
Macro average	90.99	97.46	90.33	96.65	90.54	96.33
Weighted average						

**Table 9:** Validation and testing accuracy of the proposed models.

Experiment scenario	VGG16		DenseNet201		InceptionV3		Xception	
	Valid (%)	Test (%)	Valid (%)	Test (%)	Valid (%)	Test (%)	Valid (%)	Test (%)
Feature extractor	80.64	79.36	94.57	93.81	91.63	89.73	92.11	90.99
Fine-tuner	95.21	95.25	99.23	99.71	96.92	96.78	98.12	97.92

**Table 10:** Comparison of proposed models with other deep learning models.

Models	Retinal diseases	Classification accuracy (%)
*Models proposed in the literature*		
OctNET [13]	DME, CNV, and Drusen	99.7
Layer guided CNN [35]	DME, CNV, and Drusen	89.9
GAN [16]	DME, CNV, MH and Drusen	93.9
Deep CNN [36]	DMD and DME	95.7
CenterNet [11]	DR	98.1
AlexNet, ResNet-18, GoogleNet [18]	CSR	99.6
Capsule network [22]	DME, Drusen, and CNV	99.6
CNN [24]	DMD, DME, and CNV	97.0
Deep CNN [23]	CSR	93.8

*Proposed pretrained models in this work*		
VGG16	AMD, CNV, DME, CSE, DR, Drusen, MH	
(a) As a feature extractor		79.36
(b) As a fine tuner		95.25
Densenet201		
(a) As a feature extractor		**93.81**
(b) As a fine tuner		**99.71**
InceptionV3		
(a) As a feature extractor		89.73
(b) As a fine tuner		96.78
Xception		
(a) As a feature extractor		90.99
(b) As a fine tuner		97.92

**Table 11:** Trainable parameters in proposed models.

Model	Number of parameters retrained	
	Feature extractor (M)	Fine-tuner (M)
VGG16	4.7	5.5
Xception	8.3	14.4
InceptionV3	1.1	2.3
DenseNet201	2.31	3.9

## Data Availability

The data used to support the findings of this study are included within the article.
